# Methods Used in Computer-Aided Diagnosis for Breast Cancer Detection Using Mammograms: A Review

**DOI:** 10.1155/2020/9162464

**Published:** 2020-03-12

**Authors:** Saleem Z. Ramadan

**Affiliations:** Department of Industrial Engineering, German Jordanian University, Mushaqar 11180, Amman, Jordan

## Abstract

According to the American Cancer Society's forecasts for 2019, there will be about 268,600 new cases in the United States with invasive breast cancer in women, about 62,930 new noninvasive cases, and about 41,760 death cases from breast cancer. As a result, there is a high demand for breast imaging specialists as indicated in a recent report for the Institute of Medicine and National Research Council. One way to meet this demand is through developing Computer-Aided Diagnosis (CAD) systems for breast cancer detection and diagnosis using mammograms. This study aims to review recent advancements and developments in CAD systems for breast cancer detection and diagnosis using mammograms and to give an overview of the methods used in its steps starting from preprocessing and enhancement step and ending in classification step. The current level of performance for the CAD systems is encouraging but not enough to make CAD systems standalone detection and diagnose clinical systems. Unless the performance of CAD systems enhanced dramatically from its current level by enhancing the existing methods, exploiting new promising methods in pattern recognition like data augmentation in deep learning and exploiting the advances in computational power of computers, CAD systems will continue to be a second opinion clinical procedure.

## 1. Introduction

Cancer is a disease that occurs when abnormal cells grow in an uncontrolled manner in a way that disregards the normal rules of cell division, which may cause uncontrolled growth and proliferation of the abnormal cells. This can be fatal if the proliferation is allowed to continue and spread in such a way that leads to metastasis formation. The tumor is called malignant or cancer if it invades surrounding tissues or spreads to other parts of the body [1]. Breast cancer forms in the same way and usually starts in the ducts that carry milk to the nipple or in the glands that make breast milk. Cells in the breast start to grow in an uncontrolled manner and form a lump that can be felt or detected using mammograms [2]. Breast cancer is the most prevalent cancer between women and the second cause of cancer-related deaths among them worldwide [3–5]. According to the American Cancer Society's forecasts for 2019, there will be about 268,600 new cases in the United States of invasive breast cancer diagnosed in women, about 62,930 new noninvasive cases, and about 41,760 death cases from breast cancer [3]. The death rates among women dropped 40% between 1989 and 2016, and since 2007, the death rates in younger women are steady and are steadily decreasing in older women due to early detection through screening, increased awareness, and better treatment [3, 6].

Mammography, which is performed at moderate X-ray photon energies, is commonly used to screen for breast cancer [7, 8]. If the screening mammogram showed an abnormality in the breast tissues, a diagnostic mammogram is usually recommended to further investigate the suspicious areas. The first sign of breast cancer is usually a lump in the breast or underarm that does not go after the period. Usually, these lumps can be detected by screening mammography long before the patient can notice them even if these lumps are very small to do any perceptible changes to the patient [9].

Several studies showed that using screening mammography as an early detection tool for breast cancer reduces breast cancer mortality [10–12]. Unfortunately, mammography has a low detection rate and 5% to 30% of false-negative results depending on the lesion type, the age of the patient, and the breast density [13–19]. Denser breasts are harder to diagnose as they have low contrast between the cancerous lesions and the background [20, 21]. The miss of classification in mammography is about four to six times higher in dense breasts than in nondense breasts [17, 20–24]. Dense breast reduces the test sensitivity (increases false-positive value), hence requiring unnecessary biopsy, and decreases test specificity (increases false-negative value), hence missing cancers [25].

Radiologists try to enhance the sensitivity and specificity of mammography by double reading the mammograms by different radiologists. Some authors reported that double reading enhances the specificity and sensitivity of mammography [26–28] but with extra cost on the patient. A recent study [29] and an older study [30] showed that the detection rate of double reading was not statistically different from the detection rate of a single reading in digital mammograms and hence the double reading is not a cost-effective strategy in digital mammography. The inconsistency in the results shows that there is a need for further studies in this area. Recently, Computer-Aided Diagnosis (CAD) systems are used to assist doctors in reading and interpreting medical images such as the location and the likelihood of malignancy in a suspicious lesion [7]. CADe and CADx schemes are used to differentiate between two strands of CAD systems. The main difference between CADe and CADx is that CADe stands for Computer-Aided Detection system, in which CADe systems do not present the radiological characteristics of tumors but help in locating and identifying possible abnormalities in the image and leaving the interpretation to the radiologist. On the other hand, CADx stands for Computer-Aided Diagnosis system, in which CADx serves as decision aids for radiologists to characterize findings from radiological images identified by either a radiologist or a CADe system. CADx systems do not have a good level of automation and do not detect nodules.

CAD helped the doctors to improve the interpretations of images in terms of accuracy in detection and productivity in time to read and interpret the images [31–37]. A study regarding CAD systems showed an increase in the radiologists' performance for those who used CAD systems [38]. Another study indicated that the detection rate for double reading was not significantly different from the detection rate of a single reading accompanied by a CAD system [23]. Typically, a CAD session starts with the radiologist reading the mammogram to look for suspicious patterns in it followed by the CAD system scanning the mammograms and looking for suspicious areas. Finally, the radiologist analyzes the prompts given by the CAD system about the suspicious areas [7].

The two main signs for malignancy are the microcalcification and masses [24, 39, 40]. Microcalcifications can be described in terms of their size, density, shape, distribution, and number [41]. Microcalcification detection in denser breasts is hard due to the low contrast between the microcalcification and the surrounding tissues [21]. A valuable study on how to enhance contrast, extraction, suppression of noise, and classification of microcalcification can be found in [42]. Masses, on the other hand, are circumscribed lumps in the breast and are categorized as benign or malignant. Masses can be described by shape, margin, size, location, and contrast. The shape can be further classified as round, lobular, oval, and irregular. Margin can also be further classified as obscured, indistinct, and spiculated. Masses are harder to detect by the radiologists than microcalcification because of their similarity to the normal tissues [43, 44]. Many studies presented the usage of CAD systems in mammography diagnosis such as [7, 45–50]. Like any other algorithm for a classification problem, the CAD system can be divided into three distinct areas: feature extraction, feature selection, and classification methodologies. On top of these three major areas, CAD systems depend heavily on an image enhancement step to prepare the mammogram for further analysis.  Figure 1 shows a flowchart for a typical CAD system schema.

In this study, we are presenting the developments of CAD methods used in breast cancer detection and diagnosis using mammograms, which include preprocessing and contrast enhancement, features extraction, features selection, and classification methods. The rest of the paper will be organized based on the schema in Figure 1 as follows: Section 2 presents the preprocessing and enhancement step, Section 3 discusses features selection and features extraction step, Section 4 is devoted to discussing classification through classifiers and combined classifiers, and Section 5 presents the conclusions.

## 2. Preprocessing and Contrast Enhancement

Mammograms do not provide good contrast between normal glandular breast tissues and malignant ones and between the cancerous lesions and the background especially in dense breasts [20–24, 51]. There are recognized poor contrast problems inherent to mammography images. According to the Beer-Lambert equation, the thicker the tissue is, the fewer the photons pass through it. This means that as the X-ray beam passes through normal glandular breast tissues and malignant ones in dense breast tissues, its attenuation will not differ much between the two tissues and hence there will be low contrast between normal glandular and malignant tissues [52]. Another well-known problem in mammograms is noise. Noise occurs in mammograms when the image brightness is not uniform in the areas that represent the same tissues as it supposes to be due to nonuniform photon distribution. This is called quantum noise. This noise reduces image quality especially in small objects with low contrast such as a small tumor in a dense breast. It is known that quantum noise can be reduced by increasing the exposure time. For health reasons, most of the time the radiologist prefers to decrease the exposure time for the patient at the expense of increasing the quantum noise, which will result in reducing the visibility of the mammogram. The presence of noise in a mammogram gives it a grainy appearance. The grainy appearance reduces the visibility of some features within the image especially for small objects with low contrast, which is the case for a small tumor in a dense breast [52, 53]. Because of this low-contrast problem, contrast enhancement techniques were proposed in the literature. A good review of conventional contrast enhancement techniques can be found in [54]. Unfortunately, there is no unified metrics for evaluating the performance of the preprocessing techniques to enhance the low-contrast problem and the existing evaluations are still highly subjective [55, 56].

Image enhancement usually is done by changing the intensity of the pixels for the input image [57]. The conventional histogram equalization technique for image enhancement is an attractive approach for its traceability and simplicity. The conventional histogram equalization starts by collecting statistics about the intensity of the image's pixels and formulating a histogram for the intensity levels and their frequency as in

(1) $$\begin{array}{c} H=\left[f_{i}\right], \end{array}$$

where *i* is intensity index and *f*_*i*_ is the frequency for intensity index *i*.

Using equation (1), a cumulative density function is defined as in

(2) $$\begin{array}{c} \text{CF}\left(i\right)=\sum_{i=0}^{L-1}\frac{f_{i}}{N}, \end{array}$$

where *L* is the number of intensity levels and *N* is the total number of pixels in the image. A transformation function is defined based on equation (2) to give the output image *I*_out_ as follows:

(3) $$\begin{array}{c} I_{\text{out}}\left(i\right)=I_{\min}+\left(I_{\max}-I_{\min}\right)\times \text{CF}\left(i\right), \end{array}$$

where *I*_min_ and *I*_max_ are the minimum and the maximum intensity levels of the input image, respectively.

Unfortunately, the conventional histogram equalization tends to shift the output image brightness to the middle of the allowed intensity range. To overcome this problem, subimage based histogram equalization methods were proposed in the literature where the input image is divided into subimages and the intensity for each subimage is manipulated independently. A bi-histogram equalization method discussed in [58, 59] splits the image into two subregions of high and low mean brightness based on the average intensity of all pixels and then applies the histogram equalization to each subregion independently. The mathematics of bi-histogram equalization method starts by calculating the expected value for the intensity of the input image as in

(4) $$\begin{array}{c} E\left[I_{\text{inp}}\right]=\sum_{i=0}^{L-1}i\times \frac{f_{i}}{N}. \end{array}$$

Based on *E*[*I*_inp_] , two subimages, *I*_low_ and *I*_high_, are created such that

(5) $$\begin{array}{c} EI_{\text{low}}=I_{\text{inp}}\left(i\right),\;\forall i\leq E\left[I_{\text{inp}}\right],\\ I_{\text{high}}=I_{\text{inp}}\left(i\right),\;\forall i>E\left[I_{\text{inp}}\right]. \end{array}$$

Then *I*_low_ and *I*_high_ are equalized using their corresponding range of intensities to produce two enhanced images *I*_low_enh__ and *I*_high_enh__. The enhanced output image is then constructed as the union of these two subimages. The first limitation for this method is that the original brightness can be preserved only if the original image has a symmetric intensity histogram such that the number of pixels in *I*_low_ is equal to the number of pixels in *I*_high_. If the histogram is not symmetric, the mean tends to shift toward the long tail and hence the number of pixels in each subimage will not be equal. The second limitation arises when pixels intensities tend to concentrate in a narrow range. This will be shown as peaks in the histogram and hence will generate artifacts in the output image. A third limitation is that the image may suffer from overenhancement especially if the brightness dispersion in the image is high such that there are regions of very high and very low brightness.

To overcome the limitation generated from the unequal number of pixels in the subimages, dualistic subimage histogram equalization discussed in [60] incorporated the median value as the divider threshold in the process instead of the mean to have an equal number of pixels in each subimage. This method maximizes Shannon's entropy of the output image [61]. In this method, the input image is divided into two subimages just like with equal number pixels and hence the original brightness of the input image can be preserved to some extent. To overcome the limitation generated from pixels concentrated in a narrow range, the histogram peaks are clipped prior to cumulative density calculations [62]. The procedure used is similar to bi-histogram equalization method discussed earlier in which two subimages are created along with their histograms, but on the top of that, the mean values for the two subimages are calculated as the clipping limits for the subimages as in

(6) $$\begin{array}{c} {\text{CL}}_{\text{low}}=\sum_{i=0}^{E\left[I_{\text{inp}}\right]}i\times \frac{f_{i}}{N},\\ {\text{CL}}_{\text{high}}=\sum_{i=E\left[I_{\text{inp}}\right]+1}^{L-1}i\times \frac{f_{i}}{N}. \end{array}$$

The clipping limits are used to generate the histograms for the subimages as in equation (7) and the procedure continues after that as in the bi-histogram equalization method.

(7) $$\begin{array}{c} H_{\text{low}}=\left\{\begin{array}{cc} H_{\text{low}}\left(i\right), & H_{\text{low}}\left(i\right)<{\text{CL}}_{\text{low}}\\ H_{\text{low}}, & \text{Otherwise} \end{array}\right\},\\ H_{\text{low}}=\left\{\begin{array}{cc} H_{\text{high}}\left(i\right), & H_{\text{high}}\left(i\right)<{\text{CL}}_{\text{high}}\\ H_{\text{high}}, & \text{Otherwise} \end{array}\right\}. \end{array}$$

A difficulty that sometimes arises in this method is that the mean brightness for the resulting image is hard to calculate, as it sometimes does not have a closed-form expression to evaluate it [63].

An attempt to mitigate the limitation of overenhancement is by multiple division method proposed in [63] in which dynamic quadrants histogram equalization plateau limit method divides the image into four subimages. Another attempt is by median-mean based subimage clipped histogram equalization proposed in [64], which is an enhancement for the dynamic quadrants histogram equalization plateau limit method. In this method, the mean brightness of the input image was used first to divide the input image into subimages, these subimages are then further divided using the mean brightness for the subimages, and then the peaks of the subimage histogram were clipped using median values. The minimum mean brightness error bi-histogram equalization method was used in [65], which is an exhaustive search method, to determine the best separation threshold. This method, like the subimage based histogram equalization method, cannot guarantee a match between the input and the output brightness. Another drawback of this method is that it may need a considerable amount of computational time, as it is exhaustive in nature.

A dynamic stretching strategy is adopted in [63] for contrast enhancement instead of histogram equalization with the mean or median value for the separation threshold in which the efficient golden section search approach was used to find the optimal threshold, which preserves the mean brightness in the output image. Equation (8) gives the function used for the golden section search. The golden section search method is basically searching for the mean output image intensity *E*[*I*_out_] that will minimize the absolute deviation between the output image mean intensity and the input image mean intensity *E*[*I*_inp_].

(8) $$\begin{array}{c} f\left(E\left[I_{\text{out}}\right]\right)=\left|E\left[I_{\text{inp}}\right]-E\left[I_{\text{out}}\right]\right|. \end{array}$$

There are many methods in literature to reduce the noise level in X-ray images. The traditional solution to reduce noise in X-rays images is to use a Wiener filter that computes a statistical estimate of the desired output image by filtering out the noise from the input image utilizing the second-order statistics of the Fourier decomposition [66, 67]. The Wiener filter minimizes the overall mean square error between the output image and the input image as in

(9) $$\begin{array}{c} \min\left(E\left[{\left(f\left(x,y\right)-\hat{f}\left(x,y\right)\right)}^{2}\right]\right). \end{array}$$

By taking the derivatives of equation (9), the Fourier transformation, $\hat{F}\left(u,v\right)$, of the constructed image can be derived as in

(10) F^u,v=H∗u,vH2u,v+Sζ/Sf×Gu,v,

where *f*(*x*, *y*) is the original image, $\hat{f}\left(x,y\right)$ is the constructed image, *H*^*∗*^(*u*, *v*) is the complex conjugate of the Fourier transform of the degradation filter, *H*^2^(*u*, *v*) is the momentum square of the degradation filter, *S*_*ζ*_ is the power spectrum of the noise, *S*_*f*_ is the power spectrum of the original image, *G*(*u*, *v*) is the observation, and (*H*^*∗*^(*u*, *v*)/(*H*^2^(*u*, *v*)+(*S*_*ζ*_/*S*_*f*_))) is the Wiener filter. The output image is just the input image multiplied by the Wiener filter.

The Bayesian estimator is an extension to Wiener filter to exploit the higher-order statistics found in the point statistics of the subband decomposition of natural images, which cannot be captured by Fourier based techniques [68]. The Bayesian estimator needs to have the probability density function of the noise and the prior probability density function of the signal and hence usually parametrization model is needed to estimate the parameters for those functions. Let *y* be a scalar *x* with additive noise *n* such that *y*=*x*+*n*. The least-square estimator of *x* as a function of *y* can be derived using Bayes' rule as in

(11) $$\begin{array}{c} \hat{x}\left(y\right)=\int \text{d}xP_{\left.x\right|y}\left(\left.x\right|y\right)x\\ =\hat{x}\left(y\right)=\frac{\int \text{d}xP_{\left.y\right|x}\left(\left.y\right|x\right)P_{x}\left(x\right)x}{\int \text{d}xP_{\left.y\right|x}\left(\left.y\right|x\right)P_{x}\left(x\right)}\\ =\hat{x}\left(y\right)=\frac{\int \text{d}xP_{n}\left(y-x\right)P_{x}\left(x\right)x}{\int \text{d}xP_{n}\left(y-x\right)P_{x}\left(x\right)}, \end{array}$$

where *P*_*n*_ is the *pdf* for the noise, *P*_*x*_ is the prior *pdf* for the signal, and the denominator is the *pdf* for the noise observations. Both probability density functions must be known to estimate the original signal *x*. A generalized Laplacian distribution was used by [69] as a parameterization model for these densities.

The wavelet transformation is a signal processing technique used to represent real-life nonstationary signals with high efficiency [70]. Continuous and discrete wavelet transformations are used extensively in image processing especially in microcalcification enhancement methods in mammograms [71].

Wavelet decomposes the signal into subbands using a mother wavelet function to generate other window functions. The mother wavelet function is a scaling and translation function of the form

(12) $$\begin{array}{c} \psi_{a,b}\left(x\right)=\frac{1}{\sqrt{\left|a\right|}}\psi \left(\frac{x-a}{b}\right), \end{array}$$

where *a* is the scaling factor and *b* is the translation parameters. The mother wavelet function is applied to the original function *f*(*x*) as in

(13) $$\begin{array}{c} \left(W_{\psi }f\right)\left(a,b\right)=\left\{f,\psi_{a,b}\left(x\right)\right\}=\int f\left(x\right)\cdot \psi {*}_{a,b}\left(x\right)\text{d}x. \end{array}$$

Images are 2D and hence a 2D discrete wavelet transform is needed, which can be computed using 2D wavelet filters followed by 2D downsampling operations for one level decomposition [72].

Microcalcification in mammograms was detected using a wavelet transformation with supervised learning through a cost function in [73]. The cost function represented the difference between the desired output image and the reconstructed image, which is obtained from the weighted wavelet coefficient for the mammogram under consideration. Then, a conjugate gradient algorithm was used to modify the weights for wavelet coefficients to minimize the cost function. In [74], the continuous wavelet transform was used to enhance the microcalcification in mammograms. In this method, a filter bank was constructed by discretizing a continuous wavelet transform. This discrete wavelet decomposition is designed in an optimal way to enhance the multiscale structures in mammograms. The advantage of this method is that it reconstructs the modified wavelet coefficients without the introduction of artifacts or loss of completeness.

Reference [75] presented a tumor detection system for fully digital mammography that detects the tumor with very weak contrast with its background using iris adaptive filter, which is very effective in distinguishing rounded opacities regardless of how weak its contrast with the background. The filter uses the orientation map of gradient vectors. Let *Q*_*i*_ be any arbitrary pixel and let *g* be gradient vector toward the pixel of interest *P*; then, the convergence index can be expressed as

(14) $$\begin{array}{c} f\left(Q_{i}\right)=\left\{\begin{array}{cc} \cos\theta , & \left|g\right|\neq 0\\ 0, & \left|g\right|=0 \end{array}\right\}, \end{array}$$

where *θ* is the orientation of the gradient vector *g* at *Q*_*i*_ with respect to the *i*th half line. The average of convergence indexes over the length *PQ*_*i*_, i.e., *C*_*i*_ is calculated by

(15) $$\begin{array}{c} C_{i}=\frac{\int_{P}^{Q_{i}}f\left(Q\right)\text{d}Q}{PQ_{i}}. \end{array}$$

The output of the iris filter *C*(*x*, *y*) at the pixel (*x*, *y*) is given by equation (16), where *C*_*im*_ is the maximum convergence degree deduced from equation (15):

(16) $$\begin{array}{c} C\left(x,y\right)=\frac{1}{N}\sum_{i=0}^{N-1}C_{im}. \end{array}$$

Reference [54] lists a number of other contrast enhancement algorithms with their advantages and limitations. For example, manual intensity windowing is limited by its operator skill level. Histogram-based intensity windowing has the advantage of improving the visibility of the lesion edge but at the expense of losing the details outside the dense area of the image. Mixture-model intensity windowing enhances the contrast between the lesion borders and the fatty background but at the expense of losing mixed parenchymal densities near the lesion. Contrast-limited adaptive histogram equalization improves the visibility of the edges but at the expense of increasing noise. Unsharp masking improves visibility for lesion's borders but at the expense of misrepresenting indistinct masses as circumscribed. Peripheral equalization represents the lesion details well and keeps the peripheral details of the surrounding breast but at the expense of losing the details of the nonperipheral portions of the image. Trex processing increases visibility for lesion details and breast edges but at the expense of deteriorating image contrast.

## 3. Feature Selection and Feature Extraction

Pattern, as described in [76], is the opposite of chaos, i.e., regularities. Pattern recognition is concerned with automatic discovering of these regularities in data utilizing computer algorithms in order to take action like classification under supervised or unsupervised setup [77, 78]. Pattern recognition has been studied in various frameworks but the most successful framework is the statistical framework [79–82]. A good reference for discussing statistical tools for features selection and features extraction can be found in [83]. In a statistical framework, a pattern is described by a vector of *d* features in *d*-dimensional space. This framework aims to reduce the number of features used to allow the pattern vector, which belongs to different categories, to occupy compact and disjoint regions in *m*-dimensional feature space to improve classification, stabilize representation, and/or to simplify computations [78]. A preprocessing and contrast step, which includes outlier removal, data normalization, handling of missing data, and enhancing contrast, is usually performed before the selection and extraction step [84]. The effectiveness of the selection step is measured by how successful the different patterns can be separated [76]. The decision boundaries between the patterns are determined by the probability distributions of the patterns belonging to the corresponding class. These probability distributions can be either provided or learned [85, 86]. Because selecting an optimal subset of features is done offline, having an optimal subset of features is more important than execution time [85].

The selection step involves finding the most useful subset of features that best classifies the data into the corresponding categories by reducing the *d*-dimensional features vector into an *m*-dimensional vector such that *m* ≤ *d* [84]. This can be done by features selection in measurement space (i.e., features selection) or transformation from the measurements to lower-dimensional feature space (i.e., features extraction). Features extraction can be done through a linear or nonlinear combination of the features and can be done under supervision or no supervision [83]. The most important features that are usually extracted from the mammograms are *spectral* features, which correspond to the variations in the quality of color and tone in an image; *Textural* features, which describe the spatial distribution of the color and tone within an image, and *contextual* features, which contain the information from the area surrounding the interest region [67]. Textural features are very useful in mammograms and can be classified into fine, coarse, or smooth, rippled, molled, irregular, or lineated [67]. Several linear and nonlinear features extraction techniques based on textural features are used in mammograms analysis such as in [72, 87–95].

Considering *M* classes and corresponding feature vectors distributed as *p*(*x*|*w*_*i*_), the parametric likelihood functions, and the corresponding parameters vectors *θ*_*i*_, we can find the corresponding probability density function *p*(*x*|*θ*_*i*_). A maximum log-likelihood estimator, or other methods like Bayesian inference, can be used to estimate the unknown parameters giving the set of known feature vectors. The expected maximization algorithm can be used to handle missing data. Having the probability density functions for the data available, we can extract meaningful features from them.

Gray-level cooccurrence matrix (GLCM) proposed by [67] is a well-established method for texture features extraction and is used extensively in the literature [80, 96–104]. Fourteen features were extracted from GLCM by the same author who originally proposed it [105]. The basic idea of the GLCM is as follows: let *I* be an *N*-greyscale level image, and then the gray-level cooccurrence matrix *G* for *I* is an *N* square matrix with its entries being defined as the number of occasions a pixel with intensity *i* is adjacent (on its vertical, horizontal, right, or left diagonals) to a pixel with intensity *j*. The features are calculated on each possible combination of adjacency and then the average is taken. *G* can be normalized by dividing each element of *G* by the total number of cooccurrence pairs in *G*. For example, consider the following gray-level image:

(17) $$\begin{array}{c} \left[\begin{array}{ccccc} 0 & 0 & 0 & 1 & 2\\ 1 & 1 & 0 & 1 & 1\\ 2 & 2 & 1 & 0 & 0\\ 1 & 1 & 0 & 2 & 0\\ 0 & 0 & 1 & 0 & 1 \end{array}\right]. \end{array}$$

If we apply the rule “1 pixel to the right and 1 pixel down,” the corresponding gray-level cooccurrence matrix is

(18) $$\begin{array}{c} C=\frac{1}{16}\left[\begin{array}{ccc} 4 & 2 & 1\\ 2 & 3 & 2\\ 0 & 2 & 0 \end{array}\right]. \end{array}$$

For example, the first entry comes from the fact that there are 4 occasions where a 0 appears below and to the right of another 0, whereas the normalization factor (1/16) comes from the fact that there are 16 pairs entering into this matrix.

The 14 Haralick's texture features are contrast, correlation, sum of squares, homogeneity, sum average, sum variance, sum entropy, entropy, difference variance, difference entropy, information measure of correlation 1, information measure of correlation 2, and maximum correlation coefficient. Probably the most used are energy, entropy, contrast, homogeneity, and correlation [105].

Let *P*(*i*, *j*, *d*, *θ*) denote the probability of how often one gray-tone *i* in an *N*-greyscale level image will appear in a specified spatial relationship determined by the direction *θ* and the distance *d* to another gray-tone *j* in a mammogram. The probability can be calculated as

(19) $$\begin{array}{c} P\left(i,j,d,\theta \right)=\frac{C\left(i,j\right)}{\sum_{i,j=0}^{N-1}C\left(i,j\right)}, \end{array}$$

where *C*(*i*, *j*) are the values in cell (*i*, *j*).

This definition will be used to define five of the most commonly used measures of the 14 Haralick's texture features: energy, entropy, contrast, homogeneity, and correlation.

Energy, also known as angular second moment, measures the homogeneity of the image such that if the texture of the image is uniform, there will be very few dominant gray-tone transitions and hence the value of energy will be high. The energy can be calculated as

(20) $$\begin{array}{c} \text{energy}=\sum_{i,j=0}^{N-1}P^{2}\left(i,j,d,\theta \right). \end{array}$$

Entropy measures the nonuniformity in an image or complexity of an image. Entropy is strongly but inversely correlated to energy and can be calculated from the second-order histogram as

(21) $$\begin{array}{c} \text{entropy}=-\sum_{i,j=0}^{N-1}P\left(i,j,d,\theta \right)\times \log\;P\left(i,j,d,\theta \right). \end{array}$$

Contrast measures the variance of the gray level in the image, i.e., the local gray-level variations present in an image. It detects disorders in textures. For smooth images, the contrast value is low, and for coarse images, the contrast value is high.

(22) $$\begin{array}{c} \text{contrast}=\sum_{i,j=0}^{N-1}{\left(i-j\right)}^{2}\times P\left(i,j,d,\theta \right). \end{array}$$

Homogeneity, which is also known as inverse difference moment, is a measure of local homogeneity and it is inversely related to contrast such that if contrast is low, the homogeneity is high. Homogeneity is calculated as

(23) $$\begin{array}{c} \text{homogeneity}=\sum_{i,j=0}^{N-1}\frac{P\left(i,j,d,\theta \right)}{i+{\left|i-j\right|}^{2}}. \end{array}$$

Correlation is used to measure the linear dependencies in the gray-tone level between two pixels.

(24) $$\begin{array}{c} \text{Corr}=\sum_{i,j=0}^{N-1}\frac{\left(i-\mu_{x}\right)\times \left(j-\mu_{y}\right)\times P\left(i,j,d,\theta \right)}{\sigma_{x}\times \sigma_{y}}, \end{array}$$

where *μ*_*x*_ is the mean value of pixel intensity *i*, *σ*_*x*_ is the standard deviation value of pixel intensity *i*, *μ*_*y*_ is the mean value of pixel intensity *j*, and *σ*_*y*_ is the standard deviation value of pixel intensity *j*.

Figure 2 shows the mdb028 mammogram (a) from the MIAS database [106] and the corresponding region of interest (b).

The corresponding contrast, correlation, energy, entropy, and homogeneity values calculated based on the GLCM matrix are 0.0813, 0.9617, 0.2656, 6.53, and 0.9594, respectively. One can see that this image has high homogeneity and low contrast as expected.

Gradient-based methods are widely used in analyzing mammograms [107–109]. The basic idea of the gradient is as follows: let *Y* be an ℝ-valued random variable, and then

(25) $$\begin{array}{c} \frac{\partial }{\partial x}E\left[\left.Y\right|X=x\right]=B\int {\left.y\frac{\partial }{\partial z}\tilde{p}\left(\left.y\right|z\right)\right|}_{z=B^{T}x}\text{d}y, \end{array}$$

where (*X*, *Y*) is a random vector such that *X*=(*X*^1^,…,  *X*^*m*^) ∈ *ℝ*^*m*^, and *B* is a projection matrix, such that *B*^*T*^*B*=*I*_*d*_, into *d*-dimensional subspace such that *d* ≤ *m*. Equation (25) implies that the gradient ∂/∂*xE*[*Y* *|* *X*=*x*] at any *x* is contained in the effective direction for regression.

Traditional gradient methods often could not reveal a clear-cut transition or gradient information because malignant lesions usually fill a large area in the mammogram [110]. This limitation was addressed by [95] where directional derivatives were used to measure variations in intensities. This method is known as acutance, *A*, and is calculated as

(26) $$\begin{array}{c} A=\frac{\sum_{i=1}^{N}\sqrt{\sum_{j=0}^{n_{i}=1}{\left(f_{i}\left(j\right)-f_{i}\left(j+1\right)\right)}^{2}}}{f_{\max}-f_{\min}}, \end{array}$$

where *f*_max_ and *f*_min_ are the local maximum and minimum pixel values in the region under consideration, respectively, *N* is the number of pixels along the boundary of the region, and *f*_*i*_(*j*), *j*=0,1,…, *n*_*i*_ are (*n*_*i*_+1) number of perpendicular pixels available at the *i*th boundary point including the boundary point [110].

The evaluation of the spiculations of the tumor's edges through pattern recognition techniques is widely used among scholars to classify masses into malignant and benign [87, 89, 111–114]. Morphological features can help in distinguishing between benign and malignant masses. Benign masses are characterized by smooth, circumscribed, macrolobulated, and well-defined contours, while malignant masses are vague, irregular, microlobulated, and spiculated contours. Based on these morphological features of the mass, scholars defined certain measures and indicators to classify the masses into benign and malignant like the degree of compactness, the spiculation index, the fractional factor, and fractal dimension [115].

Differential analysis is also used to compare the prior mammographic image with the most current one to find if the suspicious masses have changed in size or shape. The relative gray level is also compared between the old mammogram and the current one to deduce the changes in the breast since the last mammogram by comparing the cumulative histograms of prior and current images [90]. The bilateral analysis is also used to compare the left and right mammograms to see any unusual differences between the left and right breasts [116].

The classification metrics for a classifier depends on the interrelation between sample size, number of features, and type of classifier [78]. For example, in naïve table-lookup, the number of training data points increases exponentially with the number of features [117]. This phenomenon is called the curse of dimensionality and it leads to another phenomenon. As [78] argued that as long as the number of training samples is arbitrarily large and representative of the underlying densities, the probability of misclassification of a decision rule does not increase as the number of features increases because under this condition the class-conditional densities are completely known. In practice, it has been observed that adding features will degrade the metrics of the classifier if the size of the training data used is small compared to the number of features. This inconsistent behavior is known as the peaking phenomenon [118–120]. The peaking phenomenon can be explained as follows: most of the parametric classifiers estimate the unknown parameters for the classifier and then plug them into the class-conditional densities. At the same sample size, as the number of features increases (consequently the number of unknown parameters increases), the estimation of the parameters degrades, and consequently, this will degrade the metrics of the classifier [78]. Because of the curse of dimensionality and peaking phenomena, features selection is an important step to enhance the overall metrics of the classifier. Many methods have been discussed in the literature for features selection [78, 83]. Class separability measure can help in a deep understanding of the data and in determining the separability criterion of various features classes along with suggestions for the appropriate classification algorithms.

Class separability measures are based on conditional probability. Given two classes *C*_*i*_ and *C*_*j*_ and a features vector *v*, *C*_*i*_ will be chosen if the ratio between *P*(*C*_*i*_ *|* *v*), and *P*(*C*_*j*_ *|* *v*) is more than 1. The distance *D*_*ij*_ between *C*_*i*_ and *C*_*j*_ can be calculated as

(27) $$\begin{array}{c} D_{ij}=\int_{-\infty }^{\infty }p\left(\left.v\right|C_{i}\right)\ln\frac{p\left(\left.v\right|C_{i}\right)}{p\left(\left.v\right|C_{j}\right)}\text{d}v. \end{array}$$

And *D*_*ji*_ can be calculated in the same way. The total distance *d*_*ij*_ is a measure of separability for multiclass problems. This distance is referred to as divergence or Kullback-Leibler distance measure. Kullback-Leibler distance can be calculated as discussed in [84, 121] as

(28) $$\begin{array}{c} d_{ij}=D_{ij}+D_{ji}=\int_{-\infty }^{\infty }\left(p\left(\left.v\right|C_{i}\right)-p\left(\left.v\right|C_{j}\right)\right)\ln\frac{p\left(\left.v\right|C_{i}\right)}{p\left(\left.v\right|C_{j}\right)}\text{d}v. \end{array}$$

Another well-known distance is Mahalanobis distance. Consider two Gaussian distributions with equal covariance matrices; then, the Mahalanobis distance is calculated as

(29) $$\begin{array}{c} d_{ij}={\left(\mu_{i}-\mu_{j}\right)}^{T}\Sigma^{-1}\left(\mu_{i}-\mu_{j}\right), \end{array}$$

where Σ is the covariance matrix for the two Gaussian distributions and *μ*_*i*_ and *μ*_*j*_ are their two means.

Class separability measures are important if many features are used. If up to 3 features, the analyst can see the class scatter. Three class separability measures are widely used: class scatter measure, Thornton's separability index, and direct class separability measure [122].

In class scatter measure, an unbounded measure *J* is defined as the ratio of the *between*-class scatter and the *within*-class scatter such that the larger the value of *J* is, the smaller the within-class scatter compared to the between-class scatter is. *J* can be calculated as

(30) $$\begin{array}{c} J=\frac{\sum_{i=1}^{C}{\left(m_{i}-m\right)}^{t}\left(m_{i}-m\right)}{\sum_{i=1}^{C}\sum_{j=1}^{n_{i}}{\left(x_{ij}-m_{i}\right)}^{t}\left(x_{ij}-m_{i}\right)}, \end{array}$$

where *C* is the number of classes, *n*_*i*_ is the number of instances in class *i*, *m*_*i*_ is the mean of instances in class *i*, *m* is the overall mean of all classes, and *x*_*ij*_ is the *j*th instance in class *i*.

Separability index (SI) reports the average number of instances that share the same class label as their nearest neighbors. SI is calculated as

(31) $$\begin{array}{c} \text{SI}=\frac{\sum_{i=1}^{n}\left(f\left(x_{i}\right)+f\left(\overset{´}{x_{i}}\right)+1\right)\mathrm{mod}2}{n}. \end{array}$$

Direct class separability DCSM takes into consideration the compactness of the class compared to its distance from the other class. DCSM can be calculated as

(32) $$\begin{array}{c} \text{DCSM}=\left[\sum_{i=1}^{n_{i}}\sum_{j=1}^{n_{j}}\left\|x_{i}-x_{j}\right\|-\sum_{i=1}^{n_{i}}\sum_{i=1}^{n_{i}}\left\|x_{i}-x_{j}\right\|\right], \end{array}$$

where *x*_*i*_ and *x*_*j*_ are the instances in classes *i* and *j*, respectively.

Class separability measures aim to choose the best set of features to increase the metrics of the classifier. Without this insight choice of features, two different datasets can look alike if the features were selected in the wrong way. This phenomenon is known as Ugly Duckling Theorem [123]. Many methods are used in literature to select features and can be categorized into three main methods: filter methods, wrapper methods, and hybrid methods (which is composed of both the filter and wrapper methods).

Filter methods assign ranks to the features to denote how useful each feature is for the classifier. Once these ranks are computed and assigned, the features set is then composed with the highest N rank features. Pearson's correlation coefficient method, as a filter method, looks at the strength of the correlation between the feature and the class of data [124]. If this correlation is strong, then this feature will be selected as it will help in separating the data and will be useful in classification. The mutual information method is another filter method. The mutual information method measures the shared information between a feature and the class of the labeled data. If there is a lot of shared information, then this feature is an important feature to distinguish between different classes in the data [125]. The relief method looks for the separation capability of randomly selected instances. It selects the nearest-class instant and the opposite-class instance and then calculates a weight for each feature. The weights are updated iteratively with each random instance. This method is known for its low computational time with respect to other methods [126]. Ensemble with the data permutation method is another filter method; the concept is to combine many weak classifiers to give a better classifier than any of the single classifiers used. The same concept is used to features selection where many weak rankings are combined to give much better ranking [127].

The general idea in wrapper methods is to calculate the efficacy for a certain set of features and to update this set until a stopping criterion is reached. A greedy forward search is an example of wrapper methods. This method calculates the efficacy of the set of features on hand and replaces the current set with this set only if its efficacy is better than the efficacy of the current set; otherwise, it keeps the current set. The greedy forward method starts with one feature and keeps adding features one at a time. The classifier is evaluated each time a new feature is added, and only if the efficacy of the classifier improved, the feature is maintained [128]. This method does not guarantee an optimal solution but it picks up the features that work best together. The exhaustive search method is considered a wrapper method. Exhaustive search features selection method, also known as the brute force method, looks for every possible combination of features and selects the combination that gives the best metrics for the classifier [128]. Of course, this can be only done within a reasonable computational time with a small number of features or if the number of possible combinations is reduced by searching certain combinations only. To see how large the number of possible combinations could be, consider a dataset with 300 features, and then the number of possible sets of features is 2^300^ ≈ 2 × 10^90^ which is a huge number. To reduce this number, we may specify that the number of features that we want is 20 features, and then the number of possible sets is 300*C*20=7.5 × 10^30^ (300 choice 20) which is much lower than the first case but still impractical in terms of computational time. If we are able somehow to reduce the 300 features into 50 features and we want to choose a set of 20 features out of them, the number of sets is 50*C*20=2.7 × 10^13^ which is still a very huge number. This illustration shows that the exhaustive search method for features selection works only when the method is highly constrained.

The principal component analysis is a widely used method for dimensionality reduction. The principal component analysis is a statistical procedure used to transfer a set of possibly correlated features into a set of linearly uncorrelated features by orthogonal transformation using eigenvalue decomposition on covariance matrices of the observed regions to determine their principal components. The transformation is carried out such that the first principal component has the highest variance, which means that it accounts for the largest amount of variability in the data, and the second principal component has the second highest variance under the constraint that it is orthogonal to all other components and so on. Principal component analysis reveals the internal structure of the data. It reveals how important each feature is in explaining the variability in the data. It simply shows the higher dimensional data space onto a shadow of lower-dimensional data space [127, 129–133].

Another method in dimensionality reduction is factor analysis. Factor analysis is a statistical method that describes variability in correlated observed factors (features) in terms of a lower number of unobserved new factors (new features). The principal component analysis is often confused with factor analysis. In fact, the two methods are slightly different. The principal component analysis does not involve any new features and it only ranks the features according to their importance in describing the data while the factor analysis involves creating new features by replacing a number of correlated features with a linear combination of them to create a new feature that does not exist originally [127].

## 4. Classification

Classification is the process of categorizing observations based on a training set of data. Classification predicts the value of a categorical variable, i.e., class of the observation, based on categorical and/or numerical variables, i.e., features. In mammograms, classification is used to predict the type of mass based on the extracted set of features. Classification algorithms can be grouped into four main groups according to their ways of calculations: frequency table based, covariance matrix based, similarity functions based, and others.

ZeroR classifier is the simplest type of frequency table classifiers that ignores the features and does classification based on the class only. The class of any observation is always the class of the majority [134, 135]. The ZeroR classifier is usually used as a baseline for benchmarking with other classifiers.

OneR classifier algorithm is another type of frequency table classifier. It generates a classification rule for each feature based on the frequency and then selects the feature that has the minimum classification error. This method is simple to construct and its accuracy is sometimes comparable to the more sophisticated classifiers with the advantage of easier results interpretation [136, 137].

Naïve Bayesian (NB) classifier is also a frequency classifier based on Bayes' theorem with a strong independence assumption between the features. NB classifier is especially useful for large datasets. Its performance sometimes outperforms the performance of the more sophisticated classifiers as discussed in [138–141]. Unlike ZeroR classifier that does not use any features in the prediction and OneR classifier that uses only one feature, the NB classifier uses all the features in the prediction.

NB classifier calculates the posterior probability of the class *c* given the set of features *X*={*x*_1_, *x*_2_,…,  *x*_*n*_ } as

(33) $$\begin{array}{c} P\left(\left.c\right|x\right)=P\left(\left.x_{1}\right|c\right)\times P\left(\left.x_{2}\right|c\right)\times \cdots \times P\left(\left.x_{n}\right|c\right)\times P\left(c\right), \end{array}$$

where *P*(*x*_*i*_|*c*) is the probability of the feature *x*_*i*_ given the class *c* and *P*(*c*) is the prior probability of the class [135]. Both probabilities can be estimated from the frequency table.

One problem facing the NB classifier is known as the zero-frequency problem. It happens when a combination of a feature and a class has zero frequency. In this case, one is added for every possible combination between features and classes, so no feature-class combination has a zero frequency.

The decision tree (DT) classifier is widely used in breast cancer classification [142–144]. The strength of DT is that it can be translated to a set of rules directly by mapping from the root nodes to the leaf nodes one by one and hence the decision-making process is easy to interpret. DT can be built based on a frequency table. It develops decision nodes and leaf nodes by repetitively dividing the dataset into smaller and smaller subsets until a stopping creation is reached or a pure class with single entry is reached. DTs can handle both categorical or numerical data. The core algorithm for DTs is called ID3, which is a top-down, greedy search algorithm with no backtracking that uses entropy and information gain to divide the subset with dependency assumption between the features [145].

Entropy was introduced in the context of features selection as one of Haralick's texture features earlier. In the ID3 algorithm, entropy has the same meaning as before and it is a measure of homogeneity in the sample. It has the same basic formula of

(34) $$\begin{array}{c} E\left(S\right)=-\sum_{x\in X}P\left(i\right)\times \log\;P\left(i\right), \end{array}$$

where *S* is the current dataset under consideration which changes at each step, *X* is the set of classes in *S*, and *P*(*i*) is the probability of class *i*, which can be estimated from the frequency table based on the dataset as the proportion of the number of elements in class *x* to the number of elements in *S*. A zero entropy for a dataset indicates a perfect classification.

Information gain is the change of entropy after a dataset is split based on a certain feature, i.e., the reduction of uncertainty in *S* after splitting it using the feature.

(35) $$\begin{array}{c} \text{IG}\left(S,F\right)=E\left(S\right)-\sum_{t\in T}p\left(t\right)E\left(t\right)=E\left(S\right)-E\left(\left.S\right|F\right), \end{array}$$

where *T* is the subsets created by splitting *S* with *F* such that *S*=∪_*t*∈*T*_*t* and *p*(*t*) is the cardinality of *t* divided by the cardinality of *S*.

Overfitting is a significant problem in DTs. Overfitting is the problem of enhancing the prediction based on the training data on the expense of the prediction based on the test data. Prepruning and postpruning are used to avoid overfitting in DTs. In prepruning, the algorithm is stopped earlier before it classifies the training set perfectly while, in postpruning, the algorithm is allowed to perfectly classify the training data but then the tree is postpruned. Postpruning is more successful than prepruning because it is hard to know when exactly to stop the growth of the tree [146].

Linear Discriminant Analysis (LDA) is widely used in analyzing mammograms [51, 147] for breast cancer. LDA is a simple classifier that sometimes produces classification that is as good as the classification of the complex classifiers. It searches for a linear combination *Z* of features *X* that best separates two classes *c*_1_ and *c*_2_ such that

(36) $$\begin{array}{c} Z=\beta_{1}x_{1}+\beta_{2}x_{2}+\cdots +\beta_{d}x_{d}, \end{array}$$

where *β*_*i*_ is the coefficient corresponding to feature *i* and *i*=1,  2,  …,  *d* and *d* is the number of features. The coefficients are determined such that the score function *S*(*β*) in equation (37) is maximized.

(37) $$\begin{array}{c} S\left(\beta \right)=\frac{\beta^{T}\mu_{1}-\beta^{T}\mu_{2}}{\beta^{T}C\beta }, \end{array}$$

where *β* is a vector of coefficients for the linear model given in equation (36) and can be calculated as

(38) $$\begin{array}{c} \beta =C^{-1}\left(\mu_{1}-\mu_{2}\right), \end{array}$$

where *μ*_1_ and *μ*_2_ are the mean vectors of the two classes, and *C* is pooled covariance matrix given as

(39) $$\begin{array}{c} C=\frac{1}{n_{1}+n_{2}}\left(C_{1}n_{1}+C_{2}n_{2}\right), \end{array}$$

where *C*_1_,  *n*_1_,  *C*_2_, and *n*_2_ are covariance matrix for the first class, the number of elements in the first class, the covariance matrix for the second class, and the number of elements for the second class, respectively. A new point *x* is classified as *C*_1_, i.e., class 1, if the inequality (40) stands:

(40) $$\begin{array}{c} \beta^{T}\left(x-\left(\frac{\mu_{1}+\mu_{2}}{2}\right)\right)>-\log\frac{P\left(C_{1}\right)}{P\left(C_{2}\right)}, \end{array}$$

where *P*(*C*_1_) is the first-class probability and *P*(*C*_2_) is the probability of the second class. These probabilities can be estimated from the data.

The logistic regression classifier is another covariance classifier that is used to analyze mammograms for breast cancer prediction [148–151]. It can be used only with binary classification where there are only two classes just like classifying the masses into benign or malignant in a mammogram. It uses categorical and/or numerical features to predict a binary variable (the class either 0 or 1). Linear regression is not appropriate to predict a binary variable because the residuals will not be normal and the linear regression may predict values outside the permissible range, i.e., 0 to 1 while logistic regression can only produce values between 0 and 1 [152].

Logistic regression uses the natural logarithm of the odds of the class variable. The logistic regression equation is written in terms of the odd ration as in

(41) $$\begin{array}{c} \frac{p}{1-p}=\exp\left(b_{0}+b_{1}x_{1}+b_{2}x_{2}+\cdots +b_{n}x_{n}\right), \end{array}$$

where *p* is the logistic model predicted probability, and *b*_0_, *b*_1_,…, *b*_*n*_ are the estimations of the coefficients in the logistic regression model for the *n* features, i.e., *x*'s [151, 153]. The estimation of the model coefficients is carried out using maximum likelihood estimation. The predicted probability *p* by the logistic model can be calculated as

(42) $$\begin{array}{c} p=\frac{1}{1+e^{-\left(b_{0}+b_{1}x_{1}+b_{2}x_{2}+\cdots +b_{p}x_{p}\right)}}. \end{array}$$

One way to do classification is to calculate *p* for the data instance, and if its probability is below 0.5, it will be assigned to class 1, and if it is above or equal to 0.5, it will be assigned to class 2.

*K* nearest neighbors (*KNN*) classifier is used in literature to diagnose mammograms [154–157]. This classifier is a type of majority vote and a nonparametric classifier based on a similarity function. It stores all available cases and then classifies a new data instance based on its similarity to other points in the nearest *K* classes measured by distance. If *K*=1, then the new data instance will be assigned to the nearest neighbor's class. Generally speaking, increasing the number of classes, i.e., the value of *K*, increases the precision as it reduces the overall noise. Cross-validation is one way to determine the best value of *K* by using an independent dataset to validate the value of *K*. Also, the cross-validation technique can reduce the variance in the test error estimate calculations. A good practice is to have *K* between 3 and 10.

There are three well-known distance functions used in *KNN* classifier [158] for continuous features: Euclidean, Manhattan, and Minkowski distance functions. Their equations are as in

(43) $$\begin{array}{c} \text{Euclidean}=\sqrt{\sum_{i=1}^{k}{\left(x_{i}-y_{i}\right)}^{2}},\\ \text{Manhattan}=\sum_{i=1}^{k}\left|x_{i}-y_{i}\right|,\\ \text{Minkowski}={\left(\sum_{i=1}^{k}{\left(\left|x_{i}-y_{i}\right|\right)}^{q}\right)}^{1/q}, \end{array}$$

where *k* is the number of features, *x*_*i*_ is the value of feature *i* for object *x*, *y*_*i*_ is the value of feature *i* for object *y*, and *q* is the order of the Minkowski metric.

These three distances are valid for continuous features only. If the features are categorical, the Hamming distance given in equation (44) is used, which basically measures the number of mismatches between two vectors.

(44) $$\begin{array}{c} \text{Hamming}=\sum_{i=1}^{k}1_{x_{i}\neq y_{i}}. \end{array}$$

If features are mixed, then numerical features should be standardized between 0 and 1 before the distance is calculated.

There are three types of classifiers that are not based on the frequency table, covariance matrix, or similarity functions. These classifiers are support vector machines, artificial neural networks, and recently deep learning.

Support vector machines (SVM) classifier is first proposed by [159] and is used extensively in breast cancer detection and diagnosis using mammograms [160–166].

A linear SVM classifies a linearly separable data by constructing a linear hyperplane in N-dimensional feature space (N is the number of features) to maximize the margin distance between two classes [160].  Figure 3 shows a linear hyperplane for 2-dimensional feature space, the support vectors, and the marginal width for a linear SVM [167].

If the data is not linearly separable, it is mapped into higher-dimensional feature space by various nonlinear mapping functions like sigmoid and radial basis functions. The strength of the SVM classifier is that it does not need to have a priori density functions between the input and the output like some other classifiers and this is very important because, in practice, these prior densities are not known and there are not enough data to estimate them precisely.

The linear SVM classifier uses the training data to find the weight vector **w**=[*w*_1_,  *w*_2_,  …, *w*_*n*_]^*T*^ and the bias *b* for the decision function [161, 168] in

(45) $$\begin{array}{c} d\left(X,w,b\right)=\sum_{i=1}^{n}w_{i}x_{i}+b. \end{array}$$

The optimal hyperplane is the hyperplane that satisfies *d*(**X**,  **w**,  *b*)=0.

In the testing phase, a vector *y* is created such that

(46) $$\begin{array}{c} y=\text{sign}\left(d\left(X,w,b\right)\right). \end{array}$$

Equation (46) is used to classify a new point **X**_new_ such that if *y*(**X**_new_) is positive, then **X**_new_ belongs to class 1 and to class 2 otherwise.

The weight vector **w** and the bias *b* are found by minimizing the following model:

(47) $$\begin{array}{c} L_{d}\left(\alpha \right)=0.5\alpha^{T}H\alpha -f^{T}\alpha ,\\ \text{Subject to }y^{T}\alpha =0,\\ \alpha \geq 0, \end{array}$$

where *H* is the Hessian matrix given by

(48) $$\begin{array}{c} H=y_{i}y_{j}\left(x_{i}x_{j}\right), \end{array}$$

and *f* is a unit vector. The values of *α*_0*i*_ can be determined by solving the dual optimization problem in equation (47). These values are used to find the values of **w** and *b* as follows:

(49) $$\begin{array}{c} w=\sum_{i=1}^{l}\alpha_{0i}y_{i}x_{i},\\ b=\frac{1}{N}\sum_{i=1}^{N}\left(\frac{1}{y_{i}}-x_{i}^{T}w\right), \end{array}$$

where *N* is the number of support vectors.

As mentioned before, for nonlinearly separable data, the data has to be mapped to a higher-dimensional feature space first using a suitable nonlinear mapping function *φ*(*x*). A kernel function *K*(*x*_*i*_, *x*_*j*_) that maps the data into a very high-dimensional feature space is defined as

(50) $$\begin{array}{c} K\left(x_{i},x_{j}\right)=\varphi {\left(x_{i}\right)}^{T}\varphi \left(x_{j}\right), \end{array}$$

and the hyperplane is defined as

(51) $$\begin{array}{c} d\left(X\right)=\sum_{i=1}^{l}y_{i}\alpha_{i}K\left(x_{i},X\right). \end{array}$$

The SVM produced in model (47) is called a hard margin classifier. Soft margin classifier can be produced with the same model (47) but with adding an additional constraint 0 ≤ *α*_*i*_ ≤ *C*, where *C* is defined by the user. Soft margin SVM is preferred over the hard SVM to preserve the smoothness of the hyperplane [161].

One other classifier used extensively in detecting cancer in mammograms is the artificial neural network (ANN). This classifier is imitating the biological neural network, such as the brain. The biological neural network consists of a tremendous amount of connected neurons through a junction called synapses. Each neuron is connected to thousands of other neurons and receives signals from them. If the sum of these signals exceeds a certain threshold, a response is sent through the axon. ANN imitates this setup. In an ANN, the neurons are called nodes and these nodes are connected to each other. The strength of the connections is represented by weights such that the weight between two nodes represents the strength of the connection between them.  Figure 4 shows the generic structure for ANN in mammography where the network receives the features at the input nodes and provides the predicted class at the output node [169].

The inhabitation occurs when the weight is -1 and the excitation occurs when the weight is 1. Within each node's design, a transfer function is introduced [169]. The most used transfer functions are a unit step function, sigmoid function, Gaussian function, linear function, and a piecewise linear function. ANN usually has three layers of nodes: an input layer, a hidden layer, and an output layer.

ANNs have certain traits that make them suit breast cancer detection and diagnosis using mammograms. They are capable of learning complicated patterns [170, 171], they can handle missing data [172], and they are accurate classifiers [173–175]. In breast cancer detection and diagnosis using mammograms, the nodes of the input layer usually represent the features extracted from the region of interest (ROI) and the node in the output layer represents the class (either malignant or benign). The nodes of the input layer receive activation values as numeric information such that the higher the information, the greater the activation. The activation value is passed from node to node based on the weights and the transfer function such that each node sums the activation values that it receives and then modifies the sum based on its transfer function. The activation spread out in the network from the input layer nodes to the output layer node through the hidden layer where the output node represents the results in a meaningful way. The network learns through gradient descent algorithm where the error between the predicted value and the actual value is propagated backward by apportioning them to each node's weights according to the amount of this error the node is responsible for [176].

A deep learning (DL) or hierarchical learning classifier is a subset of machine learning that uses networks to simulate humanlike decision making based on the layers used in ANN. Unlike other machine learning techniques discussed until now, DL classifiers do not need features selection and extraction step as they adaptively learn the appropriate features extraction process from the input data with respect to the target output [177]. This is considered a big advantage for DL classifiers as the features selection and extraction step is challenging in most cases. For an image classification problem, the DL classifier needs three things to work properly: a large number of labeled images, neural network structure with many layers, and high computational power. It can reach high classification accuracy [178]. The most common type of DL architecture used to analyze images is Convolution Neural Network (CNN).

Different types of CNN were proposed recently to deal with breast cancer detection and diagnosis using mammograms problem [20, 166, 179–186]. For example, the VGG16 network is a deep CNN used to detect and diagnose lesions in mammograms. VGG16 consists of 16 layers with the final layer capable of detecting two kinds of lesions (benign and malignant) in the mammogram [186, 187]. VGG16 encloses each detected lesion with a box and attaches a confidence level in the predicted class for each detected lesion. Faster R-CNN is also a deep CNN used in breast cancer detection and diagnosis using mammograms. The basic Faster R-CNN is based on a convolutional neural network with an additional layer on the last convolutional layer called Region Proposal Network to detect, localize, and classify lesions. It uses various boxes with different sizes and aspect ratios to detect objects with different sizes and shapes [185]. A fast microcalcification detection and segmentation procedure utilizing two CNNs was developed in [186]. One of the CNNs was used for quick detection of candidate regions of interest and the other one was used to segment them. A context-sensitive deep neural network (DNN) is another CNN for detecting and diagnosing breast cancer using mammograms [188]. DNN takes into consideration both the local image features of a microcalcification and its surrounding tissues such that the DNN classifier automatically extracts the relevant features and the context of the mammogram. Handcraft descriptors and deep learning descriptors were used to characterize the microcalcification in mammograms [189]. The results showed that the deep learning descriptors outperformed the handcraft features. Pretrained ResNet-50 architecture and Class Activation Map technique along with Global Average Pooling for object localization were used in [190] to detect and diagnose breast cancer in mammograms. The results showed an area under the ROC of 0.96. A recent comprehensive technical review on the convolutional neural network applied to breast cancer detection and diagnosis using mammograms is found in [191].

To overcome the problem of overfitting in machine learning techniques such as DL and CNN, data augmentation techniques were used to generate artificial data by applying several transformations techniques to the actual data such as flipping, rotations, jittering, and random scaling to the actual data. Data augmentation is a very powerful method for overcoming overfitting. The augmented data represents a more complete set of data points. This will minimize the variance between the training and validation sets and any future testing sets. Data augmentation has been used in many studies along with DL and CNN such as [192–196].

It is well established among the scholars who work on the problem of breast cancer detection and diagnosis using mammograms and on classification problems in general that there is no “one size fits all” classifier. The classifier who is trained on a certain dataset and certain features space may not work with the same efficacy on other datasets. This problem is rooted in the “No Free Lunch Theorem” coined in [197]. “No Free Lunch Theorem” showed that there are no a priori differences between learning algorithms when it comes to an off-training-set error in a noise-free scenario where the loss function is the misclassification rate [197]. Therefore, each classifier has its own advantages and disadvantages based on the feature space and dataset used for learning [198]. For example, the features come in different representations like continuous, categorical, or binary variables and the features may have different physical meanings like energy, entropy, or size. Lump sums these diverse features into one features vector and then uses a single classifier that requires normalizing these features first, which is a tedious job. It may be easier to aggregate those features that share the same characteristics in terms of representation and physical meaning into several homogenous features vectors and then apply a different classifier to each vector separately. Moreover, even if the features are homogeneous in terms of representation and physical meaning but the number of features is large with a small number of training data points, then the estimation of the classifier parameters degrades as a result of the curse of dimensionality and peaking phenomena discussed earlier [118–120].

Because of this, scholars can improve their classification accuracy by combining outputs from different classifiers through a combining schema. From an implementation point of view, combination topologies can be categorized into multiple, conditional, hierarchical, or hybrid topologies [199]. For a thorough discussion of combinational topologies, one can consult [200, 201]. A combining schema includes a rule to determine when a certain classifier should be invoked and how each classifier interacts with other classifiers in the combination [78, 202]. The majority votes and weighted majority votes are two widely used combining schemas in literature. In majority votes, all classifiers have the same vote weight and the test instance will have the class that has the highest number of votes from different classifiers, i.e., the class that is predicted by the majority of the classifiers used in the combination. In majority votes, the classifiers have to be independent [78] as it has been shown that using majority votes with a combination of dependent classifiers will not improve the overall classification performance [203]. In weighted majority votes, each classifier has its own weight that will be changed according to its efficacy such that the weight will be decreased every time the classifier has a wrong class. The test instance will be classified according to the highest weighted majority class [203, 204].

Boosting and Bagging are also used to improve the accuracy of classification results. They were used successfully to improve the accuracy of the classifiers, like the DT classifier, by combining several classification results from the training data. Bagging combines classification results from different classifiers or from the same classifier using different subsets of training data, which is usually generated by bootstrapping. The main advantage of bootstrapping is to reduce the number of training datasets used. Bootstrapping resamples the same training dataset to create different training datasets that can be used with different classifiers or the same classifier. Bagging uses bootstrapping to create different datasets from one dataset. Bagging can be viewed as a voting combining technique and it has been implemented with majority voting or weighted majority voting such that the prediction is the class that has the majority votes or the weighted majority votes from different classifiers (or same classifier) with different training subsets. Bagging was used in the context of breast cancer detection using mammograms in several manuscripts like [205, 206]. Boosting technique attaches weights to different instances of training data such that lower weights are given to instances that were frequently classified correctly and higher weights for those who were frequently misclassified; therefore, these classes will be selected more frequently in the resampling to improve their performance. This is followed by another iteration of computing weights and this sequence is repeated until a termination condition is reached. The most popular version of boosting techniques is AdaBoost (stands for Adaptive Boosting) algorithm [207–209] which classifies the data instance as a weighted sum of the output of other weak classifiers. It is considered adaptive because the weights of the weak classifiers are changed adaptively based on their performance.

Table 1 shows a list of some common classifiers and their performance measures by the area under the receiver operating characteristic ROC curve registered in the respective papers where they were proposed/used.

For the sake of completeness, Table 2 shows a list of common databases used in CAD-related techniques. It should be noticed that the acquisition protocol of these databases normally must be rigorous and they are expensive.

## 5. Conclusions

In this study, we shed some light on CAD methods used in breast cancer detection and diagnosis using mammograms. We reviewed the different methods used in literature in the three major steps of the CAD system, which include preprocessing and enhancement, feature extraction, and selection and classification.

Studies reviewed in this article have shown that computer-aided detection and diagnosis of breast cancer from mammograms is limited by the low contrast between normal glandular breast tissues and malignant ones and between the cancerous lesions and the background, especially in dense breasts tissue. Moreover, quantum noise also reduces mammogram quality especially for small objects with low contrast such as a small tumor in a dense breast. The presence of noise in a mammogram gives it a grainy appearance, which reduces the visibility of some features within the image especially for small objects with low contrast. A wide range of histogram equalization techniques, among other techniques, were used in many articles for image enhancement to reduce the effect of low contrast by changing the intensity of the pixels for the input image. Different filters were proposed and used to reduce noises in mammograms such as Wiener filter and Bayesian estimator.

Morphological features were widely used by scholars to distinguish between benign and malignant masses. Benign masses are characterized by smooth, circumscribed, macrolobulated, and well-defined contours, while malignant masses are vague, irregular, microlobulated, and spiculated contours. Differential analysis was also used to compare the prior mammographic image with the most current one to find if the suspicious masses have changed in size or shape. The bilateral analysis is also used to compare the left and right mammograms to see any unusual differences between the left breast and right breast.

Table 1 gives a rough estimation of the average performance of the different CAD methods used and measured as the area under the ROC curve, which is about 0.86. This performance is encouraging but still not reliable enough to accept CAD systems as a standalone clinical procedure to detect and diagnose breast cancer using mammograms. Moreover, many results that were reported in the literature with excellent performance in cancer detection using CAD systems cannot be generalized as their analyses were conducted and tuned using a specific dataset. Therefore, unless a higher performance is reached with CAD systems by exploiting new promising methods like deep learning and higher computational power systems, CAD systems can only be used as a second opinion clinical procedure.

## Figures and Tables

**Figure 1:** Flow chart for a typical CAD system.

**Figure 2:** (a) Original mdb028 mammogram for a malignant patient. (b) The corresponding region of interest.

**Figure 3:** Support vectors, hyperplane, and marginal width with SVM [167].

**Figure 4:** Structure of ANN for typical breast cancer detection using mammogram [169].

**Table 1:** The area under the ROC for some common classification techniques for mammograms.

Method	Area under ROC
Binary decision tree [210]	0.90
Linear classifier [210]	0.90
PCA–LS SVM [211]	0.94
ANN [212]	0.88
Multiple expert system [213]	0.79
Texture measure with ANN [214]	0.87
Multiresolution texture analysis [215]	0.86
Subregion Hotelling observers [216]	0.94
Logistic regression [217]	0.81
KNN [218]	0.82
NB [219]	0.56
DL [190]	0.96
Genetic algorithms with SVM [220]	0.97

**Table 2:** List of common databases used in CAD-related techniques.

	MIAS [221]	DDSM [222]	UCSF/LLNL [223]	CALMa [224]	Banco Web [225]
Origin	UK	USA	USA	Italy	Brazil
Number of images	320	10480	198	3000	1400
File access	Free	Free	Paid	closed	Free, requires registration
Type of images	PGM	LJPEG	N/A	N/A	TIFF
